This article has been retracted.

# Clinical Influencing Factors of Acute Myocardial Infarction Based on Improved Machine Learning

**DOI:** 10.1155/2021/5569039

**Published:** 2021-03-27

**Authors:** Hongwei Du, Linxing Feng, Yan Xu, Enbo Zhan, Wei Xu

**Affiliations:** Department of Cardiology, The Second Affiliated Hospital of Harbin Medical University, Harbin 150081, China

## Abstract

At present, there is no method to predict or monitor patients with AMI, and there is no specific treatment method. In order to improve the analysis of clinical influencing factors of acute myocardial infarction, based on the machine learning algorithm, this paper uses the K-means algorithm to carry out multifactor analysis and constructs a hybrid model combined with the ART2 network. Moreover, this paper simulates and analyzes the model training process and builds a system structure model based on the KNN algorithm. After constructing the model system, this paper studies the clinical influencing factors of acute myocardial infarction and combines mathematical statistics and factor analysis to carry out statistical analysis of test results. The research results show that the system model constructed in this paper has a certain effect in the clinical analysis of acute myocardial infarction.

## 1. Introduction

At present, common cardiovascular diseases include hypertension, heart failure, coronary atherosclerosis, and myocardial infarction. Because of its high prevalence and high mortality, myocardial infarction (MI) has attracted wide attention. In recent years, the incidence of myocardial infarction and the number of deaths in China have been increasing. The incidence of MI is not strongly related to the region, but its mortality rate increases sharply with the increase of age [1], and the current trend of myocardial infarction is in the direction of young and middle-aged groups. Therefore, the prevention, detection, and treatment of myocardial infarction have become the research focus of medical experts and related scholars. Myocardial infarction is caused by ischemia of myocardial cells after obstruction of the coronary artery lumen of the cardiovascular system, which in turn causes myocardial cell necrosis. After extensive myocardial necrosis, the heart cannot work normally, causing fever, shock, heart failure, and even death.

AMI is a serious type of coronary heart disease, which is the main cause of death and disability, and its incidence is increasing rapidly in our country. In recent years, with the widespread popularity of chest pain center construction in our country, 70.8% of patients with acute ST-segment elevation myocardial infarction who arrived at the hospital within 12 hours of onset received reperfusion therapy [2], so their hospital mortality decreased significantly. As one of the most serious complications after acute myocardial infarction, mechanical complications after acute myocardial infarction are the main cause of death in patients after acute myocardial infarction, mainly heart rupture, including free wall rupture, heart aneurysm, ventricular septal perforation, and papillary muscle rupture. Cardiac rupture (CR), including free wall rupture, heart aneurysm, and papillary muscle rupture, has a lower incidence than the previous PCI era (currently about 0.2–1.7%). However, the mortality rate of patients without surgical treatment in the hospital is about 90% [3], and there is still a lack of effective prevention and treatment measures. At the same time, due to the rapid development of CR, patients often die before being diagnosed. Therefore, the incidence of heart rupture complicated by AMI may be underestimated. The occurrence of CR after AMI has two peaks: the first peak occurs within 24 hours after AMI, and the other peak occurs within one week after AMI. Because of its suddenness, rapid progress, and difficulty in treatment, clinical treatment is extremely difficult. At present, the diagnosis is mainly based on symptoms, signs, and cardiac color Doppler ultrasound. Surgical treatment is the only treatment that clearly improves the survival rate, and early VA-ECMO support before surgery may improve the prognosis of delayed surgery.

Timely and effective revascularization treatment is the key to reduce the mortality of AMI and improve its prognosis. The rescue system based on the chest pain center has played an important role in improving the timeliness of revascularization of AMI patients and reducing mortality. However, there are also cases where unnecessary revascularization therapy is performed on patients with CR, especially heart aneurysm, due to insufficient examination. This retrospective study aims to explore the risk factors for CR, so as to identify high-risk patients with CR as soon as possible, avoid inappropriate revascularization treatments, and adopt more effective management strategies to reduce their morbidity and mortality.

## 2. Related Works

Cluster analysis is a multivariate statistical method to classify research samples or indicators. This method is in the development stage and is still not perfect in theory. However, because it can solve many practical problems, it gets people's attention in many specific problems and application modeling. In particular, it is more effective when combined with other statistical methods [4]. The literature [5] summarized the problems of cluster analysis in the application process and put forward some insights into the testing method, so as to better apply the statistical method of cluster analysis. Hierarchical clustering is a multivariate statistical analysis method to study the classification of things according to the principle of “things gather together.” Hierarchical cluster analysis is often used in the analysis of small sample data. According to the multiple indicators (variables) and multiple observation data of the sample, the similarity or closeness relationship between the samples and indicators is quantitatively determined. Then, according to this, these samples or indicators are grouped into large and small groups to form a separated tree diagram or icicle diagram [6]. Its realization process is to first treat each piece of data as one type (there are *n* types) and calculate the distance between each data point according to the defined distance to form a matrix. After that, the two closest data points are combined into one category, which becomes n-1 category, and the distance or similarity between the newly generated category and the other categories is calculated to form a new distance matrix. According to the same principle as the second step, the two categories with the closest distance are merged. At this time, if the number of categories is still greater than 1, the method continues to repeat this step until all the data are merged into one category [7]. The advantages of systematic clustering are very obvious: it can cluster variables (samples) or records, the variables can be continuous or categorical variables, and the distance measurement methods and result representation methods it provides are also very rich. However, because it has to repeatedly calculate the distance, when the sample size is too large or there are many variables, the speed of the systematic clustering operation is obviously lower. Fast clustering is one of the most widely used methods of clustering analysis. This method has a small amount of calculation and rapid classification and can effectively process data with multiple indicators and large samples [8]. In the digital age, information processing problems of large samples are often involved, and the rapid clustering method shows a good application prospect and application value. In SPSS, a fast clustering process is specially provided, which facilitates the analysis and calculation work of the users, and is more conducive to the popular application of the method [9]. Fast clustering is to determine several representative samples as aggregation points, that is, the core of each category, according to a predetermined classification number. Then, the rest of the samples gather towards the condensation points and classify them one by one. While classifying, the positions of various condensation points are modified according to certain rules until the position of the condensation point changes little and the classification is reasonable [10]. Sometimes, the analyst can also manually specify the initial center position during analysis. This method is simple in principle and fast in calculation. Generally, the convergence result can be obtained after several rounds of iteration [11]. It is mostly applied to the classification of research samples, and it is used as the initial result of other classification studies, or preclassification [12]. However, in fast clustering applications, users are required to know the number of classifications required by the data in advance. Nevertheless, in the face of information that is not well understood, the classification number is difficult to determine. In addition, this method does not preanalyze and test the data. This may seriously affect the application effect of the fast clustering method and cause elephant clustering (excessive concentration of data in individual classes), distortion of data structure, and other unobjective and untrue classifications [13].

Machine learning is a multidisciplinary field, which includes artificial intelligence, computational complexity theory, probability and statistics, cybernetics, information theory, philosophy, physiology, neurobiology, and other disciplines. It is a process of system self-improvement. It started from the method research based on neuron model and function approximation theory and then developed to rule learning and decision tree learning based on symbolic calculus. After introducing the concepts of induction, interpretation, and analogy in cognitive psychology, up to the latest computational learning theory and statistical learning (including enhanced learning based on Markov process), it plays an important role in the application of related disciplines [14].

The formation of ventricular aneurysm (VA) after AMI is mainly local myocardial damage and even loss of contractility caused by large-area myocardial infarction [15]. In turn, ventricular remodeling occurs, which damages the normal geometric configuration of the ventricle, and leads to weakened, disappearing, or paradoxical movements of the local myocardium [16]. VA can be divided into true ventricular aneurysm and ventricular pseudoaneurysm according to its anatomical shape. True ventricular aneurysm refers to the myocardial tissue ischemic necrosis and loss of contractility, and connective tissue replaces the necrotic myocardium during the healing process, the formation of weak scar areas, and the formation of cystic or irregular bulging during systole or diastole. Ventricular pseudoaneurysm refers to a tumor-like structure formed by the pericardial tissue surrounding the breach, clogged by thrombus or adhesion after the ventricular wall slowly ruptures. The incidence rate is 0.1%, and the case fatality rate is as high as 48% [17], which can be confirmed by echocardiography. Once it is found, surgical treatment is required as soon as possible [18]. True ventricular aneurysms include recoverable functional aneurysms and permanent anatomical aneurysms. In addition, functional VA mostly occurs in the early stages of myocardial infarction. The myocardial cells innervated by the infarction related artery (IRA) have varying degrees of ischemia but not complete necrosis; that is, the necrotic myocardium is mixed with a large amount of stunned or hibernating myocardium, which in turn causes part of the ventricular wall motion to disappear or appear as paradoxical motion and reduces the pumping function of the heart. It can also be understood as the phenomenon of myocardial bulge in the infarct area caused by the early expansion of the left ventricle and the thinning and elongation of the ventricular wall in the infarct area after AMI [19–21]. Anatomical VA means that the fibrous connective tissue replaces the necrotic myocardium in the infarct area during the repair process, which causes the corresponding ventricular wall to become a fibrotic scar area lacking contractility. Meanwhile, its thickness is mostly 1/3 or thinner of normal ventricular wall, and ventricular wall bulge can be seen in both systole and diastole. In addition, early diagnosis and treatment of functional VA can prevent its development to anatomical VA. Studies have reported that the mortality rate of patients with VA after AMI is several times higher than that without VA. Therefore, clinicians can help improve the prognosis of AMI patients by early detection of high-risk patients who are prone to VA after AMI, and targeted enhancement of drug treatment and clinical observation.

When a computer solves a practical problem, the usual process is to describe how a given set of inputs can deduce the desired output. After that, people's task is to convert it into a series of instructions so that the computer can follow the instructions to get the desired results. However, for more complex problems, sometimes it is impossible to calculate the desired output from the given input, or the cost is too high. Therefore, these problems cannot be solved by traditional methods. One of the strategies to solve these problems is to make the computer learn the corresponding relationship between input and output functions from specified examples [22]. When there is an intrinsic function from input to output, the function is called the objective function. The estimation of the objective function output by the learning algorithm is called the solution of the learning problem [23]. In the learning model, there is another aspect of how the training data is generated and how to input it into the learner. There is a difference between batch learning and online learning. The former is to directly provide all the data to the learner at the beginning of learning. However, the latter allows the learner to learn only one example at a time and give its own estimate of the output before accepting the correct output [24]. For machine learners, there will be more and more data they are interested in, which will make the above quality measurement difficult to achieve. Even if they can find a hypothesis consistent with the training data, they may not be able to classify unseen data. Therefore, the ability to assume correct classification outside the training set is called generalization, which is exactly the attribute to be optimized [25].

## 3. K-Means Algorithms

K-means algorithm is a prototype-based objective function clustering method. What distinguishes this hard clustering algorithm is that the objective function of its optimization target is a certain distance sum from the data point to the prototype (category center), and then it uses the method of function extremum to obtain the adjustment rule of the iterative algorithm.

This article first uses the K-means clustering algorithm to cluster analysis of the current clinical impact of myocardial infarction (collecting relevant literature data as the original data) and then analyzes the specific factors.

As an algorithm that uses Euclidean distance as the similarity measure, the K-means algorithm is to find the optimal classification corresponding to a certain initial clustering center vector *V*=(*v*_1_, *v*_2_,…,*v*_*k*_)^*T*^ to make the clustering criterion function with the smallest value of the evaluation index *J*_*c*_ as the error sum-of-square criterion function. The function is defined as [26]

(1) $$\begin{array}{c} J_{c}=\sum_{i=1}^{k}\sum_{p\in C_{i}}\left\|p-M_{i}\right\|. \end{array}$$

In the formula, *p* is the space point of class *C*_*i*_, and *M*_*i*_ is the mean value of data objects in class *C*_*i*_.

As shown in Figure 1, the objective function is gradually reduced along different paths under different initial value vectors *V*_*A*_, *V*_*B*_, *V*_*C*_, and then the corresponding minimum values are found, respectively. Among them, the minimum corresponding to the two points *A* and *C* is the local minimum, and the minimum corresponding to the B point is the global minimum.

The K-means algorithm uses an iterative update method: In each iteration, the surrounding points are formed into *n* clusters according to *n* cluster centers, and the recalculated centroid of each cluster (that is, the average of all points in the cluster, that is, the geometric center) will be taken as the reference point for the next iteration. As the iteration makes the selected reference point closer and closer to the true cluster centroid, the objective function becomes smaller and smaller, and the clustering effect becomes better [27].

The algorithm flow is as follows:

(1) The algorithm gives a data set of size *n*, sets *I*=1, and selects *k* initial cluster centers:
  (2) $$\begin{array}{c} Z_{j}\left(I\right),\;j=1,2,3,\ldots ,k. \end{array}$$
(2) The algorithm calculates the distance between each data object and the cluster center:
  (3) $$\begin{array}{c} D\left(x_{i},Z_{j}\left(I\right)\right),\;i=1,2,3,\ldots ,n,j=1,2,3,\ldots ,k. \end{array}$$
If it meets
  (4) $$\begin{array}{c} D\left(x_{i},Z_{j}\left(I\right)\right)=\min\left\{D\left(x_{i},Z_{j}\left(I\right)\right),j=1,2,3,\ldots ,k\right\}, \end{array}$$
then *x*_*i*_ ∈ *w*_*k*_.
(3) The algorithm calculates the error sum-of-square criterion function *J*_*c*_:
  (5) $$\begin{array}{c} J_{c}\left(I\right)=\sum_{j=1}^{k}\sum_{k=1}^{n_{i}}{\left\|x_{k}^{\left(j\right)}-Z_{j}\left(I\right)\right\|}^{2}. \end{array}$$
(4) Judgment: if
  (6) $$\begin{array}{c} \left|J_{c}\left(I\right)-J_{c}\left(I-1\right)\right|≺\xi , \end{array}$$

then the algorithm ends; otherwise, *I*=*I*+1.

The algorithm calculates *k* new cluster centers:

(7) $$\begin{array}{c} Z_{j}\left(I\right)=\frac{1}{n}\sum_{k=1}^{n_{i}}x_{k}^{\left(j\right)},\;j=1,2,3,\ldots ,k. \end{array}$$

The algorithm returns to the second step.

The BWP indicator is based on the geometric structure of the sample and takes a sample in the data set as the research object to analyze the validity of the clustering results [28].

(8) $$\begin{array}{c} \text{BWP}\left(j,i\right)=\frac{\text{bsw}\left(j,i\right)}{\text{baw}\left(j,i\right)}=\frac{b\left(j,i\right)-w\left(j,i\right)}{b\left(j,i\right)+w\left(j,i\right)}\\ =\frac{\min_{1\leq k\leq c,k\neq j}\left(\left(1/n_{k}\right)\sum_{p=1}^{n_{k}}{\left\|x_{p}^{\left(k\right)}-x_{i}^{\left(j\right)}\right\|}^{2}\right)-\left(1/n_{j}-1\right)\sum_{q=1,q\neq i}^{n_{j}}{\left\|x_{q}^{\left(j\right)}-x_{i}^{\left(j\right)}\right\|}^{2}}{\min_{1\leq k\leq c,k\neq j}\left(\left(1/n_{k}\right)\sum_{p=1}^{n_{k}}{\left\|x_{p}^{\left(k\right)}-x_{i}^{\left(j\right)}\right\|}^{2}\right)+\left(1/n_{j}-1\right)\sum_{q=1,q\neq i}^{n_{j}}{\left\|x_{q}^{\left(j\right)}-x_{i}^{\left(j\right)}\right\|}^{2}}. \end{array}$$

In the formula, *k* and *j* represent coordinates, *x*_*i*_^(*j*)^ represents the *i*-th sample of the *j*-th category, *x*_*q*_^(*j*)^ represents the *q*-th sample of the *j*-th category, *x*_*p*_^(*k*)^ represents the *p*-th sample of the *k*-th category, *n*_*k*_ represents the number of samples in the *k*-th category, *n*_*j*_ represents the number of samples in the *j*-th category, and ‖·‖^2^ represents the squared Euclidean distance.

There are two main indicators of the K-means algorithm, namely, the intraclass tightness and the interclass tightness. It is hoped that the intraclass distance *w*(*j*, *i*) of the sample would be as small as possible. At the same time, it is hoped that the distance between the sample and the nearest neighbor cluster would be large; that is, the larger the minimum interclass distance *b*(*j*, *i*), the better. In order to combine these two factors, we use a linear combination to balance the two and make the function's goal consistent. We use the *b*(*j*, *i*)+*w*(*j*, *i*) function, that is, the cluster deviation distance baw(*j*, *i*) to evaluate the clustering results. Obviously, the larger the bsw(*j*, *i*), the better the sample clustering effect.

From the above, we can see that the BWP indicator reflects the clustering effectiveness of a single sample. The larger the BWP indicator value, the better the clustering effect of a single sample. Therefore, when we need to judge the clustering effect of data, we only need to pass the average value of the BWP indicator of the data. The larger the average value, the better the clustering effect; besides, the number of clusters corresponding to the maximum value is the optimal number of clusters. Thus, the following formula is obtained:

(9) $$\begin{array}{c} {\text{avg}}_{\text{BWP}}\left(k\right)=\frac{1}{n}\sum_{j=1}^{k}\sum_{i=1}^{n_{i}}\text{BWP}\left(j,i\right),\\ k_{\text{opt}}=\underset{2\leq k\leq n}{\arg\max}\left\{{\text{avg}}_{\text{BWP}}\right\}. \end{array}$$

In the formula, avg_BWP_(*k*) represents the average BWP index value when the data set is clustered into *k* categories, and *k*_opt_ represents the optimal number of clusters.

In the K-means algorithm, since the initial cluster centers are randomly selected, it may cause the phenomenon that samples in the same category are forcibly regarded as the initial cluster centers of the two categories. It will make the clustering result finally converge to the local optimal solution instead of the global optimal solution that we want. Therefore, the choice of the initial clustering center greatly affects the clustering effect of the K-means algorithm.

## 4. ART2 Neural Network

For any sequence of analog or binary input patterns, the ART2 network can quickly self-organize pattern recognition and clustering. The entire ART2 network includes the following main components: an attention subsystem and an orientation subsystem. The attention subsystem includes an input representation field *F*_1_ and a class representation field *F*_2_, mainly to complete the bottom-up vector competitive selection and similarity comparison. The orientation subsystem mainly cooperates with the attention subsystem to detect whether the similarity of the top-down and bottom-up vectors meets the detection standard, and take corresponding actions. The network structure of ART2 network is shown in Figure 2.

The ART2 network uses 2/3 learning rules, including *F*_1_ feature representation fields and *F*_2_ category representation fields. Among them, the *F*_1_ layer completes the preprocessing of the input vector self-normalization and noise suppression. After that, the vector is subjected to top-down adaptive filtering into *F*_2_ fields for comparison and competition, and the storage prototype or the node closest to the input mode is selected and activated. The selected node feeds back the storage mode to the *F*_1_ field through the top-down adaptive filter feedback channel. After processing, the preprocessed input mode and the feedback storage mode are sent to the orientation subsystem for processing.

The *F*_1_ feature represents the field feature and is an important part of the ART2 network. This field completes the preprocessing of external signals. Since the ART2 network can process data in real time, the preprocessing of the entire data is relatively complicated, and the structure of the entire field is also relatively complicated. The processing mainly includes vector normalization, nonlinear signal enhancement, noise suppression, and weakening process of mismatch.

As shown in Figure 2, *F*_1_ includes the upper, middle, and lower layers. These three layers use nonspecifically inhibited interneurons (indicated by large black circles in Figure 1) to perform vector normalization (unitization) for each mode. In addition, they can also perform vector normalization for each mode by highlighting the center and suppressing the surrounding parallel network.

In *F*_1_, nonlinear processing is introduced in the connections from the upper layer to the middle layer and from the lower layer to the middle layer. At the same time, in the learning process of the ART2 network, a given set of signals may contain background noise with different intensities. In *F*_1_, the combination of normalization processing and nonlinear feedback processing determines the noise criterion and enables the system to separate the signal from the noise. These processes especially enhance the STM mode of *F*_1_ and the LTM mode after learning. The degree of nonlinearity of the feedback signal function in *F*_1_ determines the degree of contrast enhancement and noise suppression.

When *F*_2_ receives the reset signal of the orientation subsystem, it inhibits the currently activated neuron, activates the second winning neuron, or selects a new category.

The *F*_1_ feature field is a very important part of the ART2 neural network, and the processing of external signals is completed in this field.

The common form of activation energy of all neurons in layer *F*_1_ and layer *r* is

(10) $$\begin{array}{c} x_{k}=\frac{J_{k}^{+}}{A+DJ_{k}^{-}}. \end{array}$$

In the above formula, *J*_*k*_^+^ is the excitation factor, *J*_*k*_^−^ is the suppression factor, *A* and *D* are constants, *I*_*i*_ is the *i*-th component of an input vector, and *a*, *b*, *c*, and *e* are constants. The function of *e* is to keep the activation energy limited when there is no input signal. *e* ≪ 1, and, generally, we set *e*=0. *y*_*j*_ is the activation energy of the j-th neuron in layer *F*_2_, and *g*(*y*) is the output function of layer *F*_2_. *f*(*x*) is a nonlinear function that suppresses small amplitude signals, and it determines the contrast enhancement characteristics of the *F*_1_ layer. *f*(*x*) is usually selected as a domain value function:

(11) $$\begin{array}{c} f\left(x\right)=\left\{\begin{array}{c} \begin{array}{cc} 0, & 0\leq x\leq \theta ,\\ x, & x\geq \theta , \end{array}\\ \left(0<\theta <1\right). \end{array}\right. \end{array}$$

The equation expressions of each layer of ART2 neural network can be expressed as follows:

(12) $$\begin{array}{c} w_{i}=I_{i}+au_{i},\\ x_{i}=\frac{w_{i}}{\left\|w\right\|},\\ v_{i}=f\left(x_{i}\right)+b\cdot f\left(q_{i}\right),\\ u_{i}=\frac{v_{i}}{\left\|v\right\|},\\ p_{i}=u_{i}+\sum_{j}g\left(y_{j}\right)z_{ij},\\ q_{i}=\frac{p_{i}}{\left\|p\right\|}. \end{array}$$

The three normalizations, respectively, suppress *x*, *u*, and *q*, and the suppression signal is equal to the modulus of the input vector, so that the activation energy values of the *x*, *u*, and *q* layers can be normalized. The realization of the entire comparison layer function mainly includes the following:

1. Suppression of noise.
2. Standardization, that is, enhancement of the important part of the input mode through contrast.
3. Comparison of bottom-up and top-down signals, which are used for reset.
4. Processing of real number data, and these numerical data can be arbitrarily close to each other.

The category layer is a competing network, and the bottom-up input calculation method is

(13) $$\begin{array}{c} T_{j}=\sum_{i}p_{i}z_{ji}. \end{array}$$

The specific form of the output function of the *F*_2_ layer is as follows:

(14) $$\begin{array}{c} g\left(Y_{j}\right)=\left\{\begin{array}{cc} d, & T_{j}=\underset{k}{\max}\left\{T_{k}\right\}\forall k,\\ 0, & \text{otherwise}. \end{array}\right. \end{array}$$

The *F*_2_ layer uses a single-live competition mechanism. Only the neuron with the largest dot product of the input vector and the connection weight will produce an output. In the above formula, {*T*_*k*_} does not include neurons that have been restarted by the reforming module recently. Therefore, the activation energy equation of the *p*-layer can be rewritten as

(15) $$\begin{array}{c} p_{i}=\left\{\begin{array}{cc} u_{i}, & F_{2}\text{ is not activated,}\\ u_{i}+dz_{ij}, & \text{Activation of the }j\text{th neuron in }F_{2}. \end{array}\right. \end{array}$$

The orientation system includes *r* layer and reforming module *ρ*. The *r* layer accepts the signal input from the *u* and *p* sublayers in the *F*_1_ comparison layer and compares the two signals. The signal from the *u* layer represents the external input mode, and the signal from the *F*_2_ layer represents the return of the stored module from the *m* layer.

The equation for layer *r* is

(16) $$\begin{array}{c} r_{i}=\frac{u_{i}+cp_{i}}{\left\|u\right\|+\left\|cp\right\|}. \end{array}$$

It can be expressed in vector form as

(17) $$\begin{array}{c} r=\frac{u+cp}{\left\|u\right\|+c\left\|p\right\|}. \end{array}$$

The reset conditions are

(18) $$\begin{array}{c} \frac{\rho }{\left\|r\right\|}>1. \end{array}$$

The above formula can be equivalent to

(19) $$\begin{array}{c} \rho >\left\|r\right\|. \end{array}$$

In the formula, *ρ* is the warning value, 0 < *ρ* ≤ 1, and ‖*r*‖ can be expressed as

(20) $$\begin{array}{c} \left\|r\right\|=\frac{{\left[1+2\left\|cp\right\|\cos\left(u,p\right)+{\left\|cp\right\|}^{2}\right]}^{2}}{1+\left\|cp\right\|}. \end{array}$$

In the formula, cos(*u*, *p*) is the cosine of vectors *u* and *p*. When the vectors *u* and *p* are parallel, it is impossible for cos(*u*, *p*)=1, ‖*r*‖=1 to reset the subsystem. This proves that as long as the output signal does not enter the *F*_2_ layer, *u*=*p* and the subsystem will not be reformed. In order to prevent the system from reorganizing the subsystem when it is not needed, there are three situations that need to be discussed:

(1) In the initialization phase of the ART2 network, the input vector needs to be learned or memorized, and there is no output signal in the *F*_2_ field. It can be seen from the above discussion that at this time *u*=*p* and the system will not be reformed.
(2) In the initialization phase of the ART2 network, the input vector needs to be learned or memorized, and the *F*_2_ field has an output signal. Since
  (21) $$\begin{array}{c} p_{i}=u_{i}+dz_{j},\;z_{j}={\left(z_{1j},z_{2j},\ldots ,z_{nj}\right)}^{t} \end{array}$$

and as long as we initialize the top-down weight *z*_*ij*_ to 0, the initial output signal of the *F*_2_ field will not affect the *F*_1_ field; *u*_*i*_=*p*_*i*_.

In the process of network learning, because

(22) $$\begin{array}{c} z_{ji}=z_{ij}=\frac{u_{i}}{1-d}\left(0<d<1\right), \end{array}$$

*z*_*ji*_ and *u* are parallel to each other. In this way, *p* and *u* are also parallel to each other, and the system will not be reformed.

Generally speaking, there are the following regulations for the constants in the ART2 neural network:

(23) $$\begin{array}{c} \left\{\begin{array}{c} a,b>0,\\ 0\leq d\leq 1,\\ 0<\theta \leq \frac{1}{\sqrt{M},}\\ 0<\rho \leq 1,\\ e\ll 1,\\ \frac{c\;d}{\left(1-d\right)}\leq 1. \end{array}\right. \end{array}$$

In the formula, when other conditions of the ART2 neural network remain unchanged, *c*  *d*/(1 − *d*) ≤ 1. The closer it is to 1, the smaller ‖*r*‖ is, and the more sensitive the ART2 neural network is to mismatches.

### 4.1. Top-Down Weight Initialization

In the above discussion, we can see that the top-down weight is *z*_*ij*_(0)=0.

### 4.2. Bottom-Up Weight Initialization

If we suppose that the *j*-th neuron in the *F*_2_ layer in the ART2 neural network remembers a certain input pattern, then

(24) $$\begin{array}{c} z_{ij}=\frac{u_{i}}{\left(1-d\right)},\\ \left\|z_{j}\right\|=\frac{\left\|u_{i}\right\|}{\left(1-d\right)}. \end{array}$$

If the system inputs a mode that is slightly different from the original storage mode and is not enough to cause reorganization, and this neuron wins the competition, the bottom-up weight coefficient needs to be modified to meet the needs of the new input mode. In this process, ‖*z*_*j*_‖ will decrease, and ‖*r*‖ will decrease. If it is stored in another neuron, the initial value of its connection weight is

(25) $$\begin{array}{c} \left\|z_{j}\left(0\right)\right\|=\frac{1}{\left(1-d\right)}. \end{array}$$

The ART2 neural network may change the winning neuron during the learning process, so the top-down weight coefficient also meets the following initialization condition:

(26) $$\begin{array}{c} \left\|z\right\|<\frac{1}{1-d}. \end{array}$$

Generally, a smaller random number can be used to initialize the weight coefficient. In addition, the following method can also be used to initialize the weights:

(27) $$\begin{array}{c} z_{ji}\left(0\right)\leq \frac{1}{\left(1-d\right)\sqrt{M}}. \end{array}$$

In the formula, *M* is the number of neurons in each sublayer of layer *F*_1_ in the ART2 neural network. The maximum value of *z*_*ji*_(0) must not be greater than $1/\left(1-d\right)\sqrt{M}$. The larger the value of *z*_*ji*_(0), the easier it is for the ART2 neural network to select neurons that are not occupied as the winning neural unit. When inputting a pattern with a large degree of mismatch, the warning coefficient is too small to cause realignment. At that time, the network would also choose an unoccupied neuron to store the current mode instead of modifying the weights on the basis of the original neuron. This operation can avoid frequent modification of the weights of the ART2 neural network structure so that the ART2 neural network can achieve a kind of stability. However, the value of *z*_*ji*_(0) cannot be too large; otherwise, even if the input mode is the same as the stored mode, the neuron may not win the competition. In this way, the system selects a new neuron to store the pattern, which results in two identical patterns being stored.

In practical applications, a value less than or equal to $1/\left(1-d\right)\sqrt{M}$ is generally selected as the initial connection weight.

## 5. Model Building

The clinical influencing factor analysis system of acute myocardial infarction constructed in this paper is based on the KNN algorithm. When *k* is large, this algorithm returns the most common value obtained by the first *k* closest training examples. From Figure 3, a very intuitive impression of the KNN algorithm can be obtained.

SVM can be regarded as a nearest neighbor classifier with only one representative point per class. Therefore, when SVM and KNN are considered at the same time, their different advantages can be used to enable the use of different classifications in different distributions. First, SVM is used as an INN classifier with only one representative point for each class. The consequence of this is that the support vector of each category may not be a good representative of the category. At this time, it can be combined with KNN. The reason is that from the principle of KNN, it can be known that it uses all support vectors as representative points, so that the classifier can improve the prediction accuracy. For example, for sample *x*, we first calculate the difference in the distance between *x* and the positive and negative support vectors *x*+ and *x*−. If the distance difference is greater than a given threshold, the classification plane is farther away from *x*, as shown by *β* in Figure 4. At this time, SVM classification can get good results. When the distance difference is less than a given threshold, the classification plane is closer to *X*, as shown by *α* in Figure 4.

The performance of the above model algorithm is verified and analyzed before the model is constructed. Figures 5 and 6 show the effect diagrams of the first category under the K-means algorithm after ART2 clustering again (statistical analysis of the number of cases within one month).

It is not difficult to see from the comparison of the two renderings that the maximum value of the sample curve in Figure 5 basically appears between 12 and 14 o'clock. Moreover, when the maximum value is used as the boundary, the power value on the left side of the maximum value increases slowly, and after reaching the maximum value, the power value decreases faster. The curve on the left is “concave” and the curve on the right is “convex.” The sample in Figure 6 is basically the same as that in Figure 5 in terms of the maximum appearance time, but the curve shape is just opposite to that in Figure 5. In Figure 6, the data changes before the maximum value is relatively rapid, and the data change rate after the maximum value is relatively slow.

For the classification of myocardial infarction clinical factors, a simple voting method is usually used, and the category or one of the categories with the most votes is the final model output. For regression problems, a simple arithmetic averaging method is usually used to arithmetically average the regression results obtained by *k* weak learners to obtain the final model output. Since the bagging algorithm performs sampling every time to train the model, its generalization ability (the ability of the learning algorithm to adapt to fresh samples) is very strong, which is very effective in reducing the variance of the model. The structure of the integrated model is shown in Figure 7.

When bootstrap sampling is performed on the sample, some of the data will not be selected (when the sample size is large enough, the rate of not being selected is about 36.8%). This part of the data will be used to test the prediction accuracy of the model (as shown in Figure 8).

When the test data is input into the model, the prediction result of each data will be obtained. The prediction result is the voting probability of the three results formed by the algorithm in the model to analyze the data, vote, and integrate the voting results. The result with the highest voting probability is the final output result of the model. The flow chart of the data test is shown in Figure 9.

The actual results of each piece of data are compared with the predicted results, and their corresponding probabilities are summarized. The model prediction results (parts) are shown in Table 1, and the corresponding chart is shown in Figure 10.

## 6. Model Effect Tests

20 sets of cases collected were experimented in the hospital; after constructing the above model system, relevant influencing factors are analyzed, and clinical cases of acute myocardial infarction are studied. The results are shown in Table 2 and Figure 11.

After that, this paper uses the model to perform multifactor analysis of influencing factors. The results are shown in Table 3 and Figure 12.

In this study, the free wall rupture group consists of more female and older patients, but the difference was not significant. However, previous domestic studies have shown that free wall rupture is more likely in male and older patients. This may be due to the small sample size in this study, which may lead to selection bias. The median time of FMC in patients with free wall rupture is shorter than that in patients with heart aneurysm, which is similar to previous studies. However, the median time from CR to death in 14 patients with free wall rupture is 1 hour, and the median time from CR to death in hospital for 5 patients with heart aneurysm is 48 hours, with the difference being significant (*P* < 0.001). The reason is that the onset of free wall rupture is more rapid, pericardial tamponade and electromechanical separation lead to rapid deterioration of hemodynamics, and the patient quickly dies within a few hours. This is also the reason why the use of IABP in patients with free wall rupture is not high. This study also found that the proportion of patients with lateral myocardial infarction is also higher, and there is no significant difference from the anterior wall AMI. In clinical practice, due to the relatively low infarct area of the lateral wall AMI, the heart function is better preserved. Compared with the anterior wall AMI, insufficient attention has been paid. It reminds us that, for high-risk patients with lateral AMI, we must be alert to the possibility of FWR. Our study also found a higher incidence of heart aneurysm in patients with anterior wall AMI (11 cases, 73.3%). The reason may be that both the anterior wall of the heart and the ventricular septum participate in blood supply through the left anterior descending branch. If the anterior descending artery is diseased, it is easy to merge with heart aneurysm in the case of anterior wall myocardial infarction. Inflammation is widely involved in myocardial repair after MI. White blood cells are involved in the removal of damaged cells and tissues. If the inflammatory response is unbalanced at this time, serious consequences such as heart rupture can occur. White blood cell count can reflect the degree of inflammation in the body. In addition, previous animal studies have also shown that inhibiting and depleting macrophages or thymosin *β*4 to reduce inflammation can reduce the incidence of CR after AMI. This study also found that increased white blood cell count is an independent risk factor for CR after AMI.

In summary, although the incidence of CR after AMI is not high, due to its high mortality, suddenness, rapid progress, and difficult treatment, sufficient attention should be paid at the beginning of the disease. At the same time, we need to confirm the diagnosis of MI in time, shorten the time from symptoms to revascularization, strengthen observation of potential CR high-risk patients, and adopt more effective management strategies to reduce their morbidity and mortality.

## 7. Conclusion

In patients with AMI, conditions such as emotional agitation, strenuous activity, and significant increase in blood pressure can induce a compensatory increase in the contractility of the normal myocardial tissue region and form shear stress between the necrotic myocardium, which can easily lead to eventual heart rupture. Therefore, it is particularly important to prevent heart rupture as early as possible through the early assessment of risk factors and active preventive methods. This article uses machine learning to analyze the clinical influencing factors of acute myocardial infarction, performing multifactor analysis through K-means algorithm, and constructs a mixed model combined with ART2 network. Moreover, this paper simulates and analyzes the model training process and builds a system structure model based on the KNN algorithm. For the classification of clinical factors of myocardial infarction, this paper uses a simple voting method, and the category with the most votes is the final model output. In addition, for regression problems, this paper uses a simple arithmetic averaging method to arithmetically average the regression results obtained by *k* weak learners to obtain the final model output. Finally, this paper uses case studies to verify the performance of the model constructed. The research results show that the model constructed in this paper has certain effects.

## Figures and Tables

**Figure 1:** Local minimum and global optimal.

**Figure 2:** Typical ART2 network structure.

**Figure 3:** Algorithm simulation diagram.

**Figure 4:** KNN model.

**Figure 5:** Clustering effect 1.

**Figure 6:** Clustering effect 2.

**Figure 7:** Integrated model structure.

**Figure 8:** Classifier model structure.

**Figure 9:** Flow chart of data test.

**Figure 10:** Statistical diagram of test results of model data.

**Figure 11:** Statistical diagram of model single factor processing.

**Figure 12:** Statistical diagram of model multifactor processing.

**Table 1:** Statistical table of test results of model data.

Number	AS = 1	AS = 2	AS = 3	Actual value	Predictive value
1	0.28820	0.68310	0.12870	2	2
2	1.09230	0.00770	0.00000	1	1
3	0.72050	0.36190	0.01870	2	2
4	1.10000	0.00000	0.00000	1	1
5	1.06370	0.03630	0.00000	2	2
6	0.24860	0.65450	0.19690	1	1
7	1.10000	0.00000	0.00000	1	1
8	0.99880	0.10010	0.00110	1	1
9	0.49830	0.53790	0.06490	3	3
10	0.10670	0.44660	0.54670	2	2

**Table 2:** Statistical table of model single factor processing.

Factor	B	Wald	*P*	OR	95% CI
Female	1.36653	9.14151	0.00303	3.90668	1.602–9.338
Age	0.0404	3.6865	0.05656	1.05141	0.999–1.085
BMI	0.02424	0.14039	0.71609	0.98576	0.861–1.107
Smoking history	0.79992	3.32896	0.06969	0.45753	0.193–1.065
History of myocardial infarction	0.42117	0.11413	0.74437	1.53318	0.133–17.382
PCI history	0.42117	0.11413	0.74437	1.53318	0.133–17.382
Hypertension	0.28785	0.43531	0.51712	0.75952	0.321–1.760
Diabetes	0.3232	0.38481	0.54237	0.73326	0.263–2.007
Hyperlipidemia	0	0	1.01	1.01	0.1–10.006
Heart failure	1.1312	0.62115	0.4343	3.1007	0.186–50.732
Arrhythmia	1.1312	0.62115	0.4343	3.1007	0.186–50.732
Cerebral infarction	0.19695	0.05151	0.83022	1.22715	0.223–6.627
White blood cell count	0.25957	16.61147	＜0.001	1.30593	1.142–1.465
Percentage of neutrophils	0.03333	1.48268	0.22826	1.04333	0.98–1.089
Hemoglobin	0.01818	3.21483	0.07474	0.99182	0.963–1.002
Platelets	0.00505	2.75831	0.09898	1.01505	0.999–1.01
Total protein	0.02929	0.86759	0.35754	0.98071	0.913–1.033
Albumin	0.04343	1.01	0.32017	0.96758	0.880–1.043
Alanine aminotransferase	0.00404	4.64802	0.03232	1.01404	1.000–1.008
Aspartate aminotransferase (U/L)	0.00606	16.82458	＜0.001	1.01606	1.003–1.009
Creatinine	0.00808	4.03798	0.04646	1.01808	1.000–1.016
Uric acid	0.00303	5.52268	0.01919	1.01303	1.001–1.006
Serum potassium	0.71205	3.60873	0.05959	2.04323	0.974–4.201
Serum sodium	0.15352	7.77902	0.00606	0.86759	0.772–0.956
Left ventricular ejection fraction (%)	0.0707	4.9288	0.02727	0.94233	0.876–0.992
Killip III-IV on admission	2.38259	20.38281	＜0.001	10.6858	3.78–29.613
Cardiogenic shock on admission	2.55934	12.80478	＜0.001	12.726	3.124–50.824
First medical contact (h)	0.00404	0.88375	0.35249	1.00596	0.989–1.004
Systolic blood pressure on admission	0.0303	7.71337	0.00606	0.98071	0.951–0.991
Diastolic blood pressure on admission	0.02222	1.74124	0.19089	0.98879	0.948–1.011
Heart rate on admission	0.04141	11.88164	0.00101	1.05242	1.018–1.066
Front wall	0.09393	0.04747	0.83729	0.92011	0.391–2.123
Sidewall	0.59489	1.11504	0.29593	1.82002	0.601–5.407
Lower wall	0	0	1.01	1.01	0.431–2.319
Back wall	1.15645	4.06121	0.04545	3.17342	1.026–9.620
Right ventricle	0	0	1.01	1.01	0.252–3.975
Left trunk	1.09585	1.93819	0.16766	2.9896	0.638–13.741
Anterior descending branch	0.26058	0.09999	0.75952	1.30694	0.261–6.423
Circumflex	0.71912	1.83214	0.17978	0.49591	0.174–1.383
Right coronary artery	0.39289	0.48177	0.4949	0.68478	0.225–2.044
Multivessel disease	0.41915	0.48985	0.49086	0.6666	0.205–2.124
IABP	2.43006	8.09717	0.00505	11.19787	2.097–58.619
PCI	1.7372	13.39159	＜0.001	0.18079	0.071–0.452
Thrombolysis	0.7373	0.60903	0.44137	2.09474	0.329–13.072
Mechanically assisted ventilation	3.53803	37.10336	＜0.001	33.55422	10.701–103.138
Beta blockers	1.79376	14.48643	＜0.001	0.17069	0.068–0.424
ACEI/ARB	2.51389	22.92397	＜0.001	0.08383	0.030–0.231
Statins	1.93617	4.58338	0.03232	0.14847	0.025–0.850
Double antiplatelet	22.56037	0	0	0	0
Aspirin	22.56037	0	0	0	0
Clopidogrel	0.42723	0.96859	0.33027	1.54227	0.654–3.564
Ticagrelor	0.65953	2.05636	0.15554	0.52621	0.212–1.276
Anticoagulant	0.193	0.195	0.659	1.213	0.514–2.861

**Table 3:** Statistical table of model multifactor processing.

Factor	*B*	Wald	*P*	OR	95% CI
Heart rate	0.03636	5.14494	0.02424	1.04737	1.004–1.071
Leukocyte	0.17473	4.16524	0.04242	1.20089	1.007–1.405
Use of beta blockers	1.94728	5.93375	0.01515	0.14645	0.032–0.692
PCI	1.70791	5.68226	0.01818	0.18584	0.047–0.746

## Data Availability

The data used to support the findings of this study are restricted. Data are available from the corresponding author for researchers who meet the criteria for access to confidential data.
